The article "Leaf Recognition Based on Joint Learning Multiloss of Multimodel Convolutional Neural Networks: A Testing for Vietnamese Herb" was published in 2021. Journal: Comput Intell Neurosci.

# Leaf Recognition Based on Joint Learning Multiloss of Multimodel Convolutional Neural Networks: A Testing for Vietnamese Herb

**DOI:** 10.1155/2021/5032359

**Published:** 2021-09-23

**Authors:** Trinh Tan Dat, Pham Cung Le Thien Vu, Nguyen Nhat Truong, Le Tran Anh Dang, Vu Ngoc Thanh Sang, Pham The Bao

**Affiliations:** Information Science Faculty, Sai Gon University, Ho Chi Minh City, Vietnam

## Abstract

A new modification of multi-CNN ensemble training is investigated by combining multiloss functions from state-of-the-art deep CNN architectures for leaf image recognition. We first apply the U-Net model to segment leaf images from the background to improve the performance of the recognition system. Then, we introduce a multimodel approach based on a combination of loss functions from the EfficientNet and MobileNet (called as multimodel CNN (MMCNN)) to generalize a multiloss function. The joint learning multiloss model designed for leaf recognition allows each network to perform its task and cooperate with the others simultaneously, where knowledge from various trained deep networks is shared. This cooperation-proposed multimodel is forced to deal with more complicated problems rather than a simple classification. Therefore, the network can learn much rich information and improve its generalization capability. Furthermore, a multiloss trade-off strategy between two deep learning models can reduce the effect of redundancy problems in ensemble classifiers. The performance of our approach is evaluated by our custom Vietnamese herbal leaf species dataset, and public datasets such as Flavia, Leafsnap, and Folio are used to build test cases. The results confirm that our approach enhances the leaf recognition performance and outperforms the current standard single networks while having less low computation cost.

## 1. Introduction

In pattern recognition field, image classification related to the labeling of input images into a fixed set of categories is challenging. This field involves various techniques for detecting and extracting features from input images and maps them with available templates in the database. Classification of natural objects such as plants and herbal species in the surrounding environments has become an important task. Recognizing valuable, threatened plants and herbal species may raise awareness among people in our society to partially contribute to preserve them.

Vietnam has rich herbal and land-plant resources that need to be preserved and efficiently exploited to promote the economic growth of high-tech agriculture. However, these valuable sources are in danger due to human activities. The information on various herbal and plant species is quite limited to nonexpert users with many barriers. Effective exploitation and conservation of precious herbal resources in Vietnam are urgent issues to be addressed, especially when the pharmaceutical market in Vietnam is currently facing serious problems, including counterfeit, low quality, and unknown sources [1]. Currently, the use of herbal products (tea, functional foods, medicines, and other forms) is becoming a new trend in the world [2]. Many consumers and patients select natural products (derived mainly from medicinal plants) because they believe these products are more compatible with the human body and have fewer side effects, and they are safe when used for a long time [3]. Therefore, we build a database on herbs and plants and recognize them with necessary information, illustrations, and urgent jobs. This information should be presented in a concise, specific manner but still ensures correctness so that mass users can easily interact with the data sources, which will be reviewed by reputable herbalists and plant experts.

The article "Leaf Recognition Based on Joint Learning Multiloss of Multimodel Convolutional Neural Networks: A Testing for Vietnamese Herb" was published in 2021. Journal: Comput Intell Neurosci.

The classification of plants and herbal species is usually distinguishable by local characteristics such as leaves, stems, roots, and fruit. It is easier to collect leaves instead of other plant organs and use them as the primary reference for plant recognition [4]. Furthermore, the morphology variations are the most observable character of a plant leading to the most effective and appreciate method for plant recognition. Therefore, leaf recognition becomes the most popular approach and plays a critical role in plant identification.

In this study, we attempt to perform leaf recognition for Vietnamese herbal leaf species. To generalize a multiloss function, we present a multimodel method based on a combination of loss functions from the EfficientNet and MobileNet. The joint learning enables each network to execute its task independently while also cooperate with the others simultaneously. Additionally, the proposed model addressed more complex issues than a simple classification.

The rest of this paper is organized as follows: in Section 2, we summarize the existing works. In Section 3, a method for the achievement of leaf recognition, for which the U-Net for leaf image segmentation is firstly introduced (Section 3.1), is proposed. The CNN and multimodel CNN are proposed for leaf recognition (Section 3.2 and 3.3).  Section 4 describes the experiment results of the proposed approach and the comparison with the other approaches. The conclusion is given in Section 5.

## 2. Literature Review

Many works reported in the literature regarding leaf recognition were motivated by the challenges from variations of shapes, various view angles, illumination effects, and various sizes [4]. These issues reduce the performance of the recognition system. The following fundamental research issues should be considered to design a realistic recognition system: feature extractor and classifier. Conventionally, these two steps in the traditional approaches such as using handcrafted feature extraction (shape-based features [5], the histogram of oriented gradients [6], and wavelet coefficients [7]) or traditional learning methods (k-nearest neighbor (KNN) [5], support vector machine (SVM) [7], random forest [8], matrix factorization framework [9], and discriminant analysis [10]) are typically computed or trained separately. As a result, errors at various steps would combine during the identifying process and be significantly affected by system performance. Moreover, building a leaf recognition system with many separated steps requires various hand-engineered domain knowledge such as feature extraction, image processing, and shape-based method knowledge. The traditional techniques make the recognition system complicated and inefficient, and they can be significantly affected by the accuracy of the recognition system. Consequently, it is not easy for nonexperts to design and develop a good-performing leaf recognition system for new applications.

The article "Leaf Recognition Based on Joint Learning Multiloss of Multimodel Convolutional Neural Networks: A Testing for Vietnamese Herb" was published in 2021. Journal: Comput Intell Neurosci.

To overcome the drawbacks of conventional recognition, the improvements in feature learning models have been driven by deep learning techniques through image classification algorithms based on the most popular labeled dataset, ImageNet [11, 12]. The new robust techniques lead to training the leaf recognition model end-to-end to simplify the above steps into a single deep learning model. The end-to-end recognition approaches reduce the complexity of the handcrafted feature extraction process in the traditional recognition system, and feature vectors are learned during the training process.

Conventionally, there has been a great variety of proposed leaf recognition algorithms. Du et al. [5] used nine digital morphological features for feature extraction. These feature vectors of training leaf images are classified by move median center (MMC) hypersphere classifier. This approach achieves good performance on a leaf dataset including 20 species of plant leaves. SVM approach can also be successfully used for plant leaf recognition. One such method combines Zernike moments and histogram of oriented gradients features and SVM for recognition [6]. The technique achieved high performance for the Flavia database and the Swedish Leaves database. Adams et al. [8] introduce a method for the recognition of medicinal plants. They collected leaves from 24 different medicinal plant species. They employed a large number of features based on the leaf shape, such as length, width, perimeter, area, and color ratio as feature extraction techniques, while random forest copes with the medical leaf recognition. In [13], the authors introduced a method for plant leaf image recognition by combining the fractal dimension and venation fractal dimension features and k-nearest neighbors. The fractal dimension of leaf edges and veins image is employed together using a projection wavelet to extract feature vectors, while the KNN copes with the classification. In [14], the authors proposed a new method based on distributed hierarchical graph neurons to extract feature vectors from various shapes of leaves in datasets. The KNN was used as the classifier. Munisami et al. [15] introduce a leaf dataset called Folio dataset for leaf recognition. The authors proposed KNN-based leaf recognition, in which shape features and color histogram are used for feature vector extraction. Chaki et al. [16] proposed a method of using a neuro-fuzzy classifier for leaf recognition. The combination of shape and texture feature from leaf images were used as input to the classifier. The curvelet transform was applied to extract information of leaf shape, and the texture is modeled using a Ridge Filter. They claimed that the feature vectors were invariant to geometric transformations.

The article "Leaf Recognition Based on Joint Learning Multiloss of Multimodel Convolutional Neural Networks: A Testing for Vietnamese Herb" was published in 2021. Journal: Comput Intell Neurosci.

However, building a traditional image classification system such as leaf recognition is quite a tricky task. It is necessary to develop a robust feature extraction for extracting rich information from leaves. This procedure requires additional domain knowledge for an efficient design. The structure of handcrafted feature extraction and classifiers are inflexible, and they need a high-quality training dataset to get significant performance. Therefore, recently researchers have focused on image classification based on convolutional neural networks (CNNs) applied to leaf recognition systems. These robust models can simultaneously learn features and build a significant classifier to overcome these drawbacks of traditional leaf recognition systems.

A promising alternative to the conventional leaf recognition systems is a deep learning framework. Recently, the leaf recognition system based on deep learning was proposed to improve the performance of the recognition system [17–20]. The CNNs have been widely and successfully used for leaf recognition. In [17], the authors developed a deep CNN-based model called LeafNet for plant species identification. They used leaf images for training and evaluating LeafNet on LeafSnap, Flavia, and Foliage datasets. Experiments on these datasets showed that the LeafNet achieves better results than handcrafted customized systems. Vilasini and Ramamoorthy [18] proposed to apply a CNN-based approach for Indian leaf species identification. The image in the dataset was taken using smartphones with white background. In this experiment, the authors used pretraining and edge detection with binary CNN to identify plant leaves more accurately. In [19], the authors identified leaves using the CNN model adjusted from the network depth using GoogleNet. They claimed that the proposed method achieved more than 94% accuracy even with leaves that have 30% damage. In addition, Sun et al. [20] presented a 26-layer ResNet for leaf recognition, which consists of 8 residual building blocks. The authors claimed that the ResNet model obtained a high accuracy.

The article "Leaf Recognition Based on Joint Learning Multiloss of Multimodel Convolutional Neural Networks: A Testing for Vietnamese Herb" was published in 2021. Journal: Comput Intell Neurosci.

It is equally important to mention that many promising methods based on multimodel/multimodal deep learning have been applied to image classification [21–27]. There are two commonly multimodel strategies: feature fusion and ensembles of multiple classifiers. In the feature fusion technique, two or more feature vectors extracted from deep learning networks are often combined by performing concatenating or averaging. The fused feature vector then is fed into a fully connected layer and softmax for classification [21–23]. This technique can obtain a better performance than conventional single networks. However, it can lead to “the curse of dimensionality” problem and does not guarantee the optimal accuracy due to the difference of feature ranges. Otherwise, combining high-level information with low-level information features can introduce the background clutter and semantic ambiguity due to the appearance of artifacts [24]. In the ensembles of multiple classifiers, each single classifier independently performs its task. Various ways of combining the output of the classifiers have been studied, such as early fusion (averaging predicted probabilities or weighted averaging) or late fusion (majority voting or weighted voting) [25–27]. It has been proved that the ensemble of multiple classifiers is generally more robust and has better performance than a single network; however, it required a large amount of computation cost and resources which are unsuitable for real-time applications with limited memory or computational resources. Furthermore, each single classifier in the ensemble technique is independently trained on data leading to the information in the trained classifier is often redundant and overlapping with each other.

This paper focuses on an approach using ensembles of deep learning architectures, called as multimodel CNN (MMCNN). To overcome the aforementioned limitations of ensemble learning, we propose to use a learning-based method by performing ensemble predictions during training, where knowledge from various trained deep networks is shared and can compress multimodel knowledge into a single one. We also introduce a multiloss trade-off strategy between two deep learning networks to reduce the effect of redundancy problems in ensemble classifiers. Furthermore, we exploit lightweight convolutional neural network architectures that achieve robust performance while using fewer parameters and FLOPS to enhance the accuracy and reduce computation cost and resources during inference task. Our main aim is to explore the effect of the CNNs, multiloss function, and ensemble learning coupled with state-of-the-art deep CNNs and their impact on leaf recognition. We first apply the U-Net model to detect and segment the leaf images from the background. We use the U-Net model as a binarization method to find the boundary of the leaf images without constraints. The U-Net was proven to be robust of segmenting objects. Next, we investigate the effect of some state-of-the-art deep CNN models for leaf recognition such as ResNet-50 V2, Xception, Inception V3, Inception-ResNet, EfficientNet, MobileNet V1, and MobileNet V2. The CNN model is used to learn informative representation directly from the input images from U-Net segmentation results. Finally, we propose a multimodel ensemble approach based on a combination of loss functions from the EfficientNet and MobileNet to general a multiloss function. In our experiments, we joint the EfficientNet and MobileNet together because these two models are small size, scaled models and have a small amount of parameters compared to the other CNN models and obtain significant accuracy experimentally. The joint learning multiloss model is suitable for leaf recognition because it allows each network to perform its task and cooperate with the other simultaneously. Under these circumstances, the proposed multimodel is forced to deal with a more complex and challenging problem rather than a simple classification. Therefore, the network can achieve generalization capability by learning rich and complex information. Moreover, we aim to build a complete ecosystem for exploiting Vietnamese herbal species' potential by constructing an online database with validated information on Vietnamese herbal species with a myriad of real captured photos. We develop a deep-learning-based approach for recognizing them based on snapshots taken by smartphones. We applied the proposed method to our custom Vietnamese herbal leaf species dataset, and public datasets such as Flavia, Leafsnap, and Folio are used to build test cases. The results confirm that the proposed approaches outperform the standard approaches in leaf recognition.

The article "Leaf Recognition Based on Joint Learning Multiloss of Multimodel Convolutional Neural Networks: A Testing for Vietnamese Herb" was published in 2021. Journal: Comput Intell Neurosci.

The contribution of this paper is described as follows:

- Build a database containing information about images of medicinal plant leaves in Vietnam. This database includes captured images of Vietnamese medicinal plants to ensure the correctness, specificity, and standards in recognize medicinal plants based on leaf features.
- Process captured images in combination with screening, removing noise, removing the background, and setting the input criteria for images (resolution, image size) by using U-Net for high accuracy in recognizing medicinal plant leaves.
- Build deep learning models based CNNs to recognize Vietnamese medicinal plant leaf based on their captured images. In addition, a MMCNN ensemble model based on joint learning multiloss is proposed to enhance the accuracy of leaf recognition. This is achieved with a two-branch CNN model by using MobileNet and EfficientNet, in which each branch enforces a specific learning loss function for learning independent discriminative capabilities. Then, a joint learning multiloss is considered to allow each branch to perform its task and also cooperate with the other at the same time, where knowledge from various trained deep networks is shared. The multiloss trade-off strategy between two deep learning models can reduce the effect of redundancy problems in ensemble classifiers.

## 3. Proposed Method

In the section, our approach is explained in detail. It includes two main steps, as shown in Figure 1. First, a preprocessing procedure is applied to remove small noise and also enhance the quality of leaf images. The preprocessing is necessary to improve the recognition. We first use the Gaussian filter to smooth the vessel image and remove small noises. Next, the U-Net convolutional network is applied to segment the boundary of leaf images and remove the background. Then, we build the CNN training and recognition architecture for segmented images from U-Net. The CNN architecture is used to automatically learn informative representations from the leaf image and make a decision. In addition, we also propose a multiloss function based on a combination of loss functions from multi-CNN models. The details of the proposed technique are described in the following sections.

### 3.1. U-Net for Leaf Image Segmentation

We use the characteristics of deep learning, namely, using the coding part of the U-Net model [28] and extracting the full connection final in training; this is a high-level feature. U-Net is one of the famous fully convolutional networks (FCNs) [29] in biomedical imaging segmentation. The FCN network has some characteristics such as upsampling operators, a successive convolutional layer, and a large number of feature channels in the upsampling part. The context information is propagated from one layer to another with higher resolution. We use architecture with U-Net segmenting leaf images from their background. This architecture consists of two parts coding and decoding. The coding part has the same architecture as the convection network model, in which the full connection layer is the last layer that the model uses to determine the results of the segmentation of input data. The U-Net model is first introduced for biomedical image segmentation, as shown in Figure 2. The network architecture includes two components, called an encoder path and a decoder path.

The article "Leaf Recognition Based on Joint Learning Multiloss of Multimodel Convolutional Neural Networks: A Testing for Vietnamese Herb" was published in 2021. Journal: Comput Intell Neurosci.

In the U-Net, the encoder is considered as a contraction path for capturing the context in input images. It is built by stacking convolutional layers followed by a rectified linear unit (ReLU), max-pooling, and dropout layers. There are two repeated convolution blocks with a kernel size of 3 × 3, each followed by a rectified linear unit (ReLU) activation function and a 2 × 2 max-pooling operation with stride 2 for downsampling. At each stage, the input dimensions are reduced by half via the max-pooling operator, while the number of feature channels is doubled. The bottleneck layer is built between the encoder and decoder path, including two 3 × 3 convolutional layers and a dropout layer. The decoder is an expansive path that is used to enable precise localization by using transposed convolutions. In the decoder, the final layer is used to map the feature vector to the binary label (i.e., leaf vs. nonleaf). The U-Net required the inputs as 2D image patches and returned the 2D segmentation probability map for each given patch. The decoder path includes an upsampling of the feature map followed by a 2 × 2 transposed convolution to recover the original dimensions of the input images and reduces half of the number of feature channels. Besides, there is a concatenation with the corresponding cropped feature channels from the encoder path and two 3 × 3 convolutional layers, each followed by a ReLU. The final layer is 1 × 1 convolution to map the feature vector to the binary prediction (i.e., leaf vs nonleaf). The configuration of U-Net architecture for leaf segmentation is shown in Table 1.

In our experiment, the original input leaf images and their corresponding segmentation maps are applied to train U-Net for extracting the boundary of leaves and remove their background. For a test case, the input image is required to the U-Net model and returns the 2D segmentation probability map. After detecting the binary map of leaves in the input image from U-Net, we apply *findContours* function in OpenCV [30] to determine the boundary of leaves in the image and then extract the rectangle around the leaf boundaries.  Figure 3 shows the results of the U-Net for leaf segmentation.

The article "Leaf Recognition Based on Joint Learning Multiloss of Multimodel Convolutional Neural Networks: A Testing for Vietnamese Herb" was published in 2021. Journal: Comput Intell Neurosci.

### 3.2. CNN Model for Leaf Recognition

The convolutional neural networks are proven effective and significant in image recognition. The CNN is built through convolutional layers, batch normalization, ReLU activation function, and max-pooling layer. We design a simple baseline CNN model for leaf recognition that consists of three convolutional layers. The first two convolutional layers are followed by a max-pooling layer, a ReLU activation, and two fully connected layers. Finally, a softmax layer is used to compute the probabilities.  Table 2 represents a simple CNN model for leaf recognition. The CNN uses convolution, max-pooling, batch normalization, and a ReLU activation function for learning features from data. Max-pooling is also used to downsample convolutional features and reduce computation cost. It enlarges the feature's corresponding time span and discards less useful features. Furthermore, batch normalization is used in the CNN layers to limit the covariate shift by fixing the means and variances of layer inputs. It enables higher learning rates, greatly accelerating the learning process, and being less careful about initialization. We use the ReLU activation function to learn the preactivation feature maps.

Furthermore, we also investigate the effective of some state-of-the-art deep CNN models for leaf recognition such as ResNet-50 V2 [31], Xception [32], Inception V3 [33], Inception-ResNet [34], EfficientNet [35], MobileNet V1 [36], and MobileNet V2 [37]. These models are used and pretrained by the ImageNet dataset. In this study, we employ the MobileNet V1 and EfficientNets B0, which are lightweight convolutional neural network architectures and achieve robust performance while using fewer parameters and FLOPS on ImageNet for leaf recognition and conducting multiloss functions. The multiloss is designed to allow each network to perform its task and cooperate with the other simultaneously. The method in this study can be deployed in low-power and limited-computing devices due to less computation.

In the MobileNet V1 architecture [36], the network is built on depthwise separable convolutions with depthwise and pointwise layers followed by batch-norm and ReLU, as shown in Figure 4. The first layer, as depthwise convolution, performs lightweight filtering via a single convolutional filter per input channel. The second layer as pointwise convolution is a 1 × 1 convolution with ReLU6, responsible for building new features based on computing linear combinations of the input channels. The ReLU6 is used as the nonlinearity because of its robustness when used with low-precision computation [36]. The MobileNet V1 architecture has 28 layers and is shown in Table 3 [36]. The standard kernels, size of 1 × 1 and 3 × 3, are applied.

The article "Leaf Recognition Based on Joint Learning Multiloss of Multimodel Convolutional Neural Networks: A Testing for Vietnamese Herb" was published in 2021. Journal: Comput Intell Neurosci.

In the MobileNet V2 network, a basic building block is represented by a bottleneck depth-separable convolution with residuals [37]. There are two types of blocks: the first one is a residual block with a stride of 1, while the second is a block with a stride of 2 for downsizing. For each type of block, there are three layers. The first layer uses 1 × 1 convolution with ReLU6. The second one is the depthwise convolution with a kernel size of 3 × 3. The last one is a linear 1 × 1 convolution. The MobileNet V2 architecture is shown in Table 4. It consists of the first initial fully convolution layer with 32 filters and 19 residual bottleneck layers. The standard kernel size of 3 × 3 is applied. Moreover, dropout and batch normalization also are used during training.

In the EfficientNets, a simple and effective compound scaling technique uses a compound coefficient *ϕ* to uniformly scale network width, depth, and resolution in a principled way [35]:

(1) $$\begin{array}{c} \text{depth}:d=\alpha^{\phi }\\ \text{width}:\;\omega =\;\beta^{\phi }\\ \text{resolution}:\;\;r=\gamma^{\phi }\\ \;s.t.\;\alpha \cdot \beta^{2}\cdot \gamma^{2}\approx 2\;,\;\alpha \geq 1,\;\beta \geq 1,\;\gamma \geq 1,\; \end{array}$$

where *ϕ* is a user-specified coefficient. It is used to control how many resources are available, while *α*, *β*, and *γ* are constants which specify how to assign these resources to network depth, width, and resolution, respectively. The EfficientNets are developed by doing a multiobjective neural architecture search that optimizes both accuracy and FLOP [35]. The architecture network is similar to M-NASNet and called as EfficientNet B0 architecture as shown in Table 5.

The main building block in the EfficientNet B0 architecture is mobile inverted bottleneck MBCon (used in MobileNet V2) with a squeeze-and-excitation optimization [35]. Based on the baseline network, we can search for optimal values for scaling parameters when *ϕ* is fixed to 1, when we fix *α*, *β*, and *γ* as constants and experiment with different values of *ϕ* as in (1) to produce EfficientNets B1-B7 [35].

### 3.3. Multiloss for Multi-CNN Model

This section proposes a new multimodel approach based on ensemble learning by using a combination of loss functions from the EfficientNet and MobileNet to general a multiloss function. In our experiments, we select the EfficientNet B0 and MobileNet V1 to conduct joint learning multiloss functions because these two models are small size, scaled models and have quite small amounts of parameters compared to the other CNN models but still obtain significant accuracy. The joint learning multiloss is proposed to suit leaf recognition. A multi-CNN model based on joint learning multiloss for leaf recognition is shown in Figure 5. In this figure, each EfficientNet and MobileNet independently performs its task, and then early fusion technique based averaging predicted probabilities to make final predictions.

The article "Leaf Recognition Based on Joint Learning Multiloss of Multimodel Convolutional Neural Networks: A Testing for Vietnamese Herb" was published in 2021. Journal: Comput Intell Neurosci.

Our model is achieved with a two-branch CNN model using MobileNet V1 and EfficientNet B0, in which each branch enforces a specific learning loss function for learning independent discriminative capabilities. Furthermore, a joint learning multiloss is then considered to allow each branch to perform its task and cooperate with the other simultaneously. The knowledge from each trained deep network is shared. The proposed multimodel is forced to deal with a more complicated problem than the simple classification. Therefore, the network is capable of learning informative features to improve the generalization. The multiloss trade-off strategy between two deep learning networks is introduced to reduce the effect of redundancy problems in ensemble classifiers.

Specifically, in our experiments, we use softmax loss or categorical cross-entropy loss to train the network to output a probability over C classes for each input. Assuming that a softmax function *f* that takes as input a given class *s*_*c*_ (*c* *=* 1,…, *C*) and outputs a *y*_*c*_ of real values between 0 and 1 is described as follows:

(2) $$\begin{array}{c} y_{c}=f{\left(s\right)}_{c}=\frac{e^{s_{c}}}{\sum_{j=1}^{C}e^{s_{j}}}\;,\;\;\text{for }c=1,\ldots ,C, \end{array}$$

where *s*_*j*_ are the scores inferred by the network for each class in *C*. The softmax loss that minimizes the negative log-likelihood is described as follows:

(3) $$\begin{array}{c} L=-\overset{C}{\underset{c=1}{\sum }}t_{c}\cdot \;\log\left(y_{c}\right), \end{array}$$

where *t*_*c*_ and *y*_*c*_ are the ground truth and the score for each class *c* in *C*.

Our multimodel approach is developed based on the idea of dividing problems into small ones and giving them to each individual in a team to solve. Assume that the multimodel is built from a combination of two models, MobileNet V1 (called HEAD1) and EfficientNet B0 (called HEAD2). The loss function of our multimodel is computed as follows:

(4) $$\begin{array}{c} \varkappa =L_{1}+L_{2}+L_{3}-3*L_{4}, \end{array}$$

where *L*_1_ denotes softmax loss between the model output and ground truth; *L*_2_ denotes softmax loss between the output of HEAD1 model and ground truth; and *L*_3_ presents softmax loss between the output of HEAD2 model and the ground truth, and *L*_4_ is cosine similarity between softmax output of models HEAD1 and HEAD2. The component *L*_1_ describes cooperation between two models HEAD1 and HEAD2 to perform recognition tasks. The components *L*_2_ and *L*_3_ orientate each model HEAD1 and HEAD2 to perform independent recognition tasks, respectively. The last term (−3*∗L*_4_) makes the most difference as possible between the two models. Finally, the multiloss function ϰ allows each model to perform its task and cooperate with the other at the same time. This can benefit from each other by exploring the relatedness, leading to boosted generalization performance.

The article "Leaf Recognition Based on Joint Learning Multiloss of Multimodel Convolutional Neural Networks: A Testing for Vietnamese Herb" was published in 2021. Journal: Comput Intell Neurosci.

## 4. Experimental Results

The experiments that were conducted to evaluate the accuracy of the leaf recognition system are presented. The information on our collected Vietnamese Herb Leaf Image Database (V-Herb database) and other public datasets is described and followed by analyzing the various parameters for evaluating the proposed approach. The experimental results of our approach are presented together with comprehensive comparisons to other studies.

### 4.1. Dataset and Analysis of the Experiments

The performance evaluation of our method is conducted on the standard three public leaf datasets such as Folio [15], Flavia [38], and Leafsnap [39] datasets. Furthermore, we also collect a leaf image database that is of Vietnamese herbal species only. The Flavia dataset contains 1907 different leaf images corresponding to 32 distinct plant species. All of the images in the Flavia leaf dataset were taken on white backgrounds. Each class has 50–77 sample images. The size of each color image is 1200 × 1600 pixels.  Figure 6 shows some images from the Flavia dataset.

The Leafsnap dataset covers 185 trees in the Northeastern United States. It contains 30866 leaf images of which are 23147 lab images and 7719 field images, respectively. The lab images are of high quality and appear in controlled environments. The fields images are taken from mobile devices at different times under varying lighting. The quality is generally worse than the quality of lab images. The size of each color image is 800 × 600 or 600 × 800 pixels. The Leafsnap dataset also includes segmentation results. The segmentation results are obtained via image processing techniques.  Figure 7 shows sample images and their segmentation results from the Leafsnap dataset. For the Folio dataset, there are 637 leaf images of 32 different species. Each class has 18–20 sample images. The size of each color image is 4128 × 2322 or 2322 × 4128 pixels. All of the images in the Folio leaf dataset were taken on a white background under varying lighting.  Figure 8 shows some images from the Folio dataset.

The article "Leaf Recognition Based on Joint Learning Multiloss of Multimodel Convolutional Neural Networks: A Testing for Vietnamese Herb" was published in 2021. Journal: Comput Intell Neurosci.

In our experiment, we use full 1907 images from the Flavia and 637 images from the Folio datasets. For the Leafsnap dataset, we only use 7552 field images from 184 different species. These field images are taken at different times with major variations, including changes in scale, rotation, and illumination. Furthermore, we combine these three datasets to evaluate the performance of the proposed method. The combination dataset (Flavia + Leafsnap + Folio) contains 239 distinct different plant species after merging and removing 09 duplicate classes. There are a total of 10057 leaf images.  Table 6 shows the information on the combination dataset in our experiment.

In addition, we are also building a Vietnamese medical leaf dataset for research. Collecting images of medicinal plants will be conducted by photographers in real environment. The collected snapshots will be screened by herbalists and plant experts. Each plant will have a separate photo folder with subdirectories divided by each section. The number of images depends on the specific requirements of each species/strain. Leaf images used in the database are of Vietnamese herbal species only. We do not use available image sources because the plants, in general, are highly variable. Their morphological feature and metabolite profiles vary according to geographical, climatic, and soil factors. The use of images captured from Vietnamese herbal species will ensure accuracy as well as noise reduction during the modeling process. The number of images and angles taken on a research object was calculated by experts to ensure the quality of input data for the model. All shooting angles must be standardized to best identify the medicinal plants. In addition, we aim to establish minimum standards for images to ensure the model can process images in the best way for high performance in recognition. At the testing, our V-Herb database obtains 373 different leaf images corresponding to 29 distinct different Vietnamese herbal species.  Table 7 shows examples of Vietnamese herbal species in our V-Herb database. All color images are taken from mobile devices on different backgrounds at different times under varying lighting conditions.  Figure 9 shows examples of leaf images in our dataset.

The performance of the U-Net approach for leaf segmentation is first described. Second, we consider the effectiveness of CNN architectures for leaf recognition. Finally, the performance of the approach based on multiloss in the multi-CNN model is compared with other well-known techniques. The CNN architectures in our experiments are implemented within the Tensorflow Keras framework. Our experiments are carried out on a computer with Intel(R) Xeon(R) CPU E5-2680 v3 @ 2.50 GHz 48 CPUs core, RTX 2080 11 VRAM, 128 GB RAM. We use the Adam optimizer with the cyclic learning rate to train our network via the backpropagation algorithm. The loss function is computed via softmax cross-entropy loss. Furthermore, we generate augmentation data for the training model. The artificially created data are performing by random transformations, such as rotation, scaling, additional brightness, flip, and blur.  Figure 10 shows examples of data augmentation in our experiments.

The article "Leaf Recognition Based on Joint Learning Multiloss of Multimodel Convolutional Neural Networks: A Testing for Vietnamese Herb" was published in 2021. Journal: Comput Intell Neurosci.

### 4.2. Segmentation Results Using U-Net

In this study, we train the U-Net on the Leafsnap dataset and the combination dataset (Leafsnap + Flavia + Folio). In the Leafsnap dataset, 7513 field leaf images with correct annotations were used for evaluating the U-Net model. There are a total of 5173 images for training, 720 images for validation, and 1620 images for testing. There are 5958 images for training in the combination dataset, 1933 images for validation, and 2166 images for testing. To training the U-Net model, we utilize the input layer as the size of 300 × 400 × 1 and the number of filters is 16.  Table 8 shows the performance of the U-Net for leaf recognition. The accuracy obtained through the U-Net is greater than 92% in the two datasets. The experimental analysis revealed that the combination dataset achieves high accuracy. So, the U-Net model has demonstrated promise for enhancing the performance of leaf image segmentation.

Figure 11 shows the comparison results of the U-Net model and binary map annotation (based on image processing techniques) on the Leafsnap dataset. This figure clearly shows that the U-Net method has achieved better accuracy than image processing techniques.  Figure 12 shows some errors of binary map annotations and output from U-Net on the Leafsnap dataset. The quality of the input images causes these errors. In these cases, some images can be affected by complex background, illumination, and noise such as low-light conditions and low contrast. These lead to reduce the accuracy of the leaf segmentation system.

Furthermore, we apply the U-Net model with pretrained on Leafsnap to perform on the Flavia dataset and with pretrained on the combination dataset to perform on our V-Herb database.  Table 9 shows the performance of U-Net segmentation for the Flavia and V-Herb database. The accuracy of U-Net segmentation on Flavia attains 100%. The U-Net model performs an accuracy of 98.63% on our dataset.

The article "Leaf Recognition Based on Joint Learning Multiloss of Multimodel Convolutional Neural Networks: A Testing for Vietnamese Herb" was published in 2021. Journal: Comput Intell Neurosci.

Experimental analysis indicated that the results on the Flavia dataset obtain very high accuracy because the images on the Flavia dataset were taken on a white background and have good quality without illumination effects.  Figure 13 presents some results of U-Net segmentation on the Flavia dataset. The U-Net model also obtains high accuracy on our dataset. Some segmentation errors occur due to the quality of the input image. In our cases, some images can be affected by illumination and noise, such as low-light conditions and low contrast. These lead to reduce the accuracy of our leaf segmentation system.  Figure 14 shows examples of U-Net segmentation results on our V-Herb database.

### 4.3. Recognition Results on Flavia Dataset

The Flavia dataset is randomly divided into 70% training, 10% validation, and 20% test dataset. We investigate the effect of U-Net combined with baseline simple CNNs for leaf recognition. To train the simple three-convolution layer CNN model in Section 3.2, we utilize the input layer as the size of 150 × 200 × 3 and the number of filters as 128. The comparative performance of leaf recognition systems is shown in Table 10.

In this table, our methods refer to U-Net + simple CNN, U-Net + VGG16, U-Net + MobileNet V1, U-Net + EfficientNet B0, and U-Net + proposed multimodel. We also compare to other methods in terms of leaf recognition. The recognition rate obtained through our methods is greater than 95% with and without data augmentation. The experimental analysis revealed that the recognition rate by using U-Net + simple CNN generally increases with applying data augmentation, with the recognition rate achieved 99.25%. However, there are certain disadvantages in increasing the computation cost. Furthermore, the U-Net + VGG16 method without data augmentation attains a 99.50% recognition rate, U-Net + MobileNet V1 obtains 100% recognition rate without data augmentation, the U-Net + EfficientNet B0 without data augmentation attains a 99.57% recognition rate, and the U-Net + proposed model without data augmentation attains a 100% recognition rate. We realize that our model yields the best accuracy on the Flavia dataset. Furthermore, without applying U-Net, our model yields a better accuracy than EfficientNet B0 and MobileNet V1 models.

The experimental results also confirm that the U-Net + proposed multimodel can enhance the recognition performance on the Flavia dataset and achieves better accuracy than other baseline CNN models. Table 10 clearly shows that the proposed method has similar or even better performance than other methods on the Flavia dataset. We consider that the Flavia dataset is simple and includes only clean images with white background, so the CNN models can obtain very high accuracy.

The article "Leaf Recognition Based on Joint Learning Multiloss of Multimodel Convolutional Neural Networks: A Testing for Vietnamese Herb" was published in 2021. Journal: Comput Intell Neurosci.

Besides, we also investigate the effect of U-Net segmentation for leaf recognition on the Flavia dataset. We compare the experiments on our simple CNN, VGG16, MobileNet V1, EfficientNet B0, and proposed multimodel with and without U-Net. Experimental analysis indicated that the simple CNN, VGG16, MobileNet V1, EfficientNet B0, and proposed model using U-Net as preprocessing yield higher accuracy than without using U-Net and are more effective than the baseline systems. The U-Net segmentation led our recognition model to work more efficiently because it helps removing unnecessary background for improving the performance of recognition.

### 4.4. Recognition Results on Combination Dataset and Our Dataset

In this section, the well-known CNN models and proposed multimodel CNN in leaf recognition systems are investigated. The combination dataset is randomly divided into 70% training, 10% validation, and 20% test. In our V-Herb database, we randomly divided it into 70% training, 5% validation, and 25% test. We also explore the effect of our multimodel CNN for leaf recognition. In the experiments, U-Net is first applied to remove background, and the output results are fed as input images to CNNs.  Table 11 shows the performance and computation cost comparison of the well-known CNNs and our proposed multimodel for leaf recognition on the combined dataset using U-Net. The recognition rate obtained through the CNNs is greater than 80% in all cases for the combination dataset. This table clearly shows that our proposed method has the best performance compared to the well-known CNN models. We realize that the multimodel CNN with multiloss significantly enhances the performance of leaf recognition. Specifically, the proposed approach obtains 93.59%. Furthermore, we also measure computation time (in average) during the inference process of our model in comparison to other single networks. From Table 11, we realize that the proposed approach-based ensemble learning performs faster than the single deep learning models as Inception-ResNet V2 and EfficientNet B2 in the term of computation cost. It only takes 0.283s to identify a single leaf image.

Furthermore, we investigate the effect of the proposed multimodel CNN on our V-Herb database.  Table 12 shows the performance and computation cost comparison of our proposed multimodel for leaf recognition on our dataset. The recognition accuracy of these systems is displayed in Table 12, which explains that the multimodel CNN-based multiloss significantly outperforms the standard CNN approaches. Particularly, the accuracy of the proposed method obtains high accuracy in the Vietnamese medical image leaf recognition. The proposed method has demonstrated a promising solution for robust performance on leaf recognition when using a multimodel approach based on multiloss function. Furthermore, there is a certain advantage with accuracy and computation cost while applied our ensemble models in comparison to other single networks. It should be noted that the modified CNN model can cope with complex problems. Thus, the multimodel network learns rich information to provide the generalization for the leaf classification.

The article "Leaf Recognition Based on Joint Learning Multiloss of Multimodel Convolutional Neural Networks: A Testing for Vietnamese Herb" was published in 2021. Journal: Comput Intell Neurosci.

Besides, we present the performance comparison in terms of accuracy for leaf recognition on our dataset with and without applying U-Net on the CNN models.  Table 13 shows comparative performance of leaf recognition with and without U-Net on our dataset. We consider that the Inception-ResNet, EfficientNet B2, and our proposed multimodel obtain a good performance compared to other models in both cases. The experiment results show that the recognition model for which the U-Net segmentation is used significantly improves the performance of the leaf recognition system and is more effective than the baseline systems because the U-Net helps to remove redundant backgrounds. Experimental analysis revealed that our proposed model achieves the best accuracy in both cases. Specifically, proposed approach attains 92.37% and 98.89% for without applying U-Net and with applying U-Net. Finally, this proves the importance of applying U-Net to increase the accuracy of the leaf recognition system.

We attribute these mistakes to the process of leaf recognition without applying U-Net segmentation. The errors often occur due to misrecognized due to unnecessary background on original image. In our dataset, leaf images are taken on large white background that includes much redundant and unnecessary information.  Figure 15 shows some leaf images taken on large background on our dataset. This leads to reduce the performance of recognition system without removing unnecessary background. Finally, the experimental results show that the recognition rate are improved significantly after removing background images.

### 4.5. Research Limitations

The primary limitation of this study is the data source. Several characteristics of herbs are not quantitatively evaluated in this study. Climate changes and local environments create herb variations in sizes, colors, and phenotypes. Generally, enriching the Vietnamese herb dataset and applying appropriate leaf quality evaluation in the preprocessing step are essential for a comprehensive analysis. Particularly, the performances of selected models are similar in Table 10 and Table 12 because of the limitation of data size and variables. However, in Table 11, the proposed model outperforms other CNN models on the combined dataset, which is considered sufficient on size and variables. It is confirmed the emergence of collect a comprehensive dataset for model comparison after a certain performance threshold. Equally important, the accuracy in Table 13 is a proof-of-concept and challenging to replicate. Firstly, the database characterizes Vietnamese local herbs, which highly depends on geographical, climatic, and soil factors. Implementing these models on different datasets will produce different results. Secondly, since the dataset is still limited in size and variances, the similar performance of selected models is reasonable. When several models archive the same performance on a dataset, it is suggested the improvement of the herb dataset in terms of size, seasons, and variables.

The article "Leaf Recognition Based on Joint Learning Multiloss of Multimodel Convolutional Neural Networks: A Testing for Vietnamese Herb" was published in 2021. Journal: Comput Intell Neurosci.

The processing time is the secondary limitation in this study. Although the proposed model requires 0.220 seconds on average for classification, this period is not good enough for real-time applications. An upgrade on hardware is a short-term solution, while further research is required as a sustainable solution.

## 5. Conclusion

We propose an improved leaf recognition technique by investigating a combination of loss functions from multimodel CNNs for joint learning multiloss tasks based on ensemble learning. In addition, the U-Net model is introduced for leaf segmentation for enhancing the performance of the overall system. The effect of the joint learning multiloss task is considered to improve leaf recognition. The experimental results prove that the proposed approach can significantly improve the accuracy and provide robust performance compared to the standard CNN methods. Our approach is effective and robust under illumination environments. Furthermore, we consider that leaf vein is one of the most important and useful features of leaf. This feature can be used in identification of plant species. In the future, we will investigate the effect of leaf vein features. We will consider a combination between the features of leaf vein and shape to enhance performance of leaf recognition systems. Besides, we will consider an exploration of the effect of graph CNN architecture in leaf recognition.

## Figures and Tables

**Figure 1:** An illustration of the proposed method for the leaf recognition.

**Figure 2:** An illustration of the U-Net architecture [28].

**Figure 3:** Results of U-Net for leaf segmentation.

**Figure 4:** A depthwise separable convolution in the MobileNet V1 model [37].

The article "Leaf Recognition Based on Joint Learning Multiloss of Multimodel Convolutional Neural Networks: A Testing for Vietnamese Herb" was published in 2021. Journal: Comput Intell Neurosci.

**Figure 5:** A multimodel CNNs based on joint learning multiloss for leaf recognition.

**Figure 6:** Some images from the Flavia dataset.

**Figure 7:** Sample images from the Leafsnap dataset.

**Figure 8:** Sample images from the Folio dataset.

**Figure 9:** Examples of leaf images in our V-Herb database.

**Figure 10:** Examples of data augmentation in our experiment.

**Figure 11:** Some comparison results of the U-Net model and binary map annotation on the Leafsnap.

**Figure 12:** Some errors in segmentation results on the Leafsnap.

**Figure 13:** Examples of U-Net segmentation on the Flavia dataset.

**Figure 14:** Examples of U-Net segmentation on our V-Herb database.

**Figure 15:** Some leaf images with large background on our dataset.

**Table 1:** The U-Net architecture for leaf segmentation.

	Layer	Size	Previous layers
Input	*input*_1	*m* × *n* × 3	

**Encoder path**	conv2d_1	*m* × *n* × *f*	input_1
	conv2d_2	*m* × *n* × *f*	conv2d_1
	maxpooling2d_1	*m*/2 × *n*/2 × *f*	conv2d_2
	conv2d_3	*m*/2 × *n*/2 × 2*f*	maxpooling2d_1
	conv2d_4	*m*/2 × *n*/2 × 2*f*	conv2d_3
	maxpooling2d_2	*m*/2^2^ × *n*/2^2^ × 2*f*	conv2d_4
	conv2d_5	*m*/2^2^ × *n*/2^2^ × 3*f*	maxpooling2d_2
	conv2d_6	*m*/2^2^ × *n*/2^2^ × 3*f*	conv2d_5
	maxpooling2d_3	*m*/2^3^ × *n*/2^3^ × 3*f*	conv2d_6
	conv2d_7	*m*/2^3^ × *n*/2^3^ × 4*f*	maxpooling2d_3
	conv2d_8	*m*/2^3^ × *n*/2^3^ × 4*f*	conv2d_7
	dropout_1	*m*/2^3^ × *n*/2^3^ × 4*f*	conv2d_8
	maxpooling2d_4	*m*/2^4^ × *n*/2^4^ × 4*f*	dropout_1

**Decoder path**	conv2d_9	*m*/2^4^ × *n*/2^4^ × 5*f*	maxpooling2d_4
	conv2d_10	*m*/2^4^ × *n*/2^4^ × 5*f*	conv2d_9
	dropout_2	*m*/2^4^ × *n*/2^4^ × 5*f*	conv2d_10
	upsampling2d_1	*m*/2^3^ × *n*/2^3^ × 5*f*	dropout_2
	cropping2d_1	*m*/2^3^ × *n*/2^3^ × 5*f*	dropout_1
	concatenate_1	*m*/2^3^ × *n*/2^3^ × 9*f*	upsampling2d_1cropping2d_1
	conv2d_11	*m*/2^3^ × *n*/2^3^ × 9*f*	concatenate_1
	conv2d_12	*m*/2^3^ × *n*/2^3^ × 4*f*	conv2d_11
	upsampling2d_2	*m*/2^2^ × *n*/2^2^ × 4*f*	conv2d_12
	cropping2d_2	*m*/2^2^ × *n*/2^2^ × 3*f*	conv2d_6
	concatenate_2	*m*/2^2^ × *n*/2^2^ × 7*f*	upsampling2d_2cropping2d_2
	conv2d_13	*m*/2^2^ × *n*/2^2^ × 3*f*	concatenate_2
	conv2d_14	*m*/2^2^ × *n*/2^2^ × 3*f*	conv2d_13
	upsampling2d_3	*m*/2 × *n*/2 × 3*f*	conv2d_14
	cropping2d_3	*m*/2 × *n*/2 × 2*f*	conv2d_4
	concatenate_3	*m*/2 × *n*/2 × 5*f*	upsampling2d_3cropping2d_3
	conv2d_15	*m*/2 × *n*/2 × 2*f*	concatenate_3
	conv2d_16	*m*/2 × *n*/2 × 2*f*	conv2d_15
	upsampling2d_4	*m* × *n* × 2*f*	conv2d_16
	cropping2d_4	*m* × *n* × *f*	conv2d_2
	concatenate_4	*m* × *n* × 3*f*	upsampling2d_4cropping2d_4
	conv2d_17	*m* × *n* × *f*	concatenate_4
	conv2d_18	*m* × *n* × *f*	conv2d_17

**Output**	conv2d_19	*m* × *n* × 3	conv2d_18

*m* × *n* denotes size of the input image; *f* denotes number of filters.

The article "Leaf Recognition Based on Joint Learning Multiloss of Multimodel Convolutional Neural Networks: A Testing for Vietnamese Herb" was published in 2021. Journal: Comput Intell Neurosci.

**Table 2:** A simple CNN architecture for leaf recognition.

	Layer	Size	Previous layer
Input	*input*_1	*m* × *n* × 3	
	conv2d_1	*m* × *n* × *f*	input_1
	maxpooling2d_1	*m*/2 × *n*/2 × *f*	conv2d_1
	conv2d_2	*m*/2 × *n*/2 × 2*f*	maxpooling2d_1
	maxpooling2d_2	*m*/2 × *n*/2 × 2*f*	conv2d_2
	conv2d_3	*m*/6 × *n*/6 × 3*f*	maxpooling2d_2

**Output**	flatten_1	*m*/6 × *n*/6 × 3*f*	conv2d_3
	dense_1	2*f*	flatten_1
	dense_2	*N*	dense_1

*m* × *n* denotes size of the input image; *f* denotes number of filters.

**Table 3:** Overall architecture of the MobileNet V1 [36].

Type/stride	Filter shape	Input size
Conv/s2	3 × 3 × 3 × 32	224 × 224 × 3
Conv dw/s1	3 × 3 × 3 dw	112 × 112 × 32
Conv/s1	1 × 1 × 32 × 64	112 × 112 × 32
Conv dw/s2	3 × 3 × 64 dw	112 × 224 × 64
Conv/s1	1 × 1 × 64 × 128	56 × 56 × 64
Conv dw/s1	3 × 3 × 128 dw	56 × 56 × 128
Conv/s1	1 × 1 × 128 × 128	56 × 56 × 128
Conv dw/s2	3 × 3 × 128 dw	56 × 56 × 128
Conv/s1	1 × 1 × 128 × 256	56 × 56 × 128
Conv dw/s1	3 × 3 × 256 dw	28 × 28 × 256
Conv/s1	1 × 1 × 256 × 256	28 × 28 × 256
Conv dw/s2	3 × 3 × 256 dw	28 × 28 × 256
Conv/s1	1 × 1 × 256 × 512	14 × 14 × 256
5 × Conv dw/s1	3 × 3 × 512 dw	14 × 14 × 512
Conv/s1	1 × 1 × 512 × 512	14 × 14 × 512
Conv dw/s2	3 × 3 × 512 dw	14 × 14 × 512
Conv/s1	1 × 1 × 512 × 1024	7 × 7 × 512
Conv dw/s2	3 × 3 × 1024 dw	7 × 7 × 1024
Conv/s1	1 × 1 × 1024 × 1024	7 × 7 × 1024
Avg Pool/s1	Pool 7 × 7	7 × 7 × 1024
FC/s1	1024 × 1000	1 × 1 × 1024
Softmax/s1	Classifier	1 × 1 × 1000

**Table 4:** Overall architecture of the MobileNet V2.

Input	Operator	*t*	*c*	*n*	*s*
224^2^ × 3	conv2d	—	32	1	2
112^2^ × 32	bottleneck	1	16	1	1
112^2^ × 16	bottleneck	6	24	2	2
56^2^ × 24	bottleneck	6	32	3	2
28^2^ × 32	bottleneck	6	64	4	2
14^2^ × 64	bottleneck	6	96	3	1
14^2^ × 96	bottleneck	6	160	3	2
7^2^ × 160	bottleneck	6	320	1	1
7^2^ × 320	conv2d 1 × 1	—	1280	1	1
7^2^ × 1280	avgpool 7 × 7	—	—	1	—
1 × 1 × 1280	conv2d 1 × 1	—	k	—	

*t* denotes expansion factor, *c* is number of output channels, *n* describes repeating number, and *s* is stride; 3 × 3 kernels are used for spatial convolution [37].

**Table 5:** Overall architecture of the EfficentNet-B0 network.

Stage *i*	Operator ${\hat{ℱ}}_{i}$	Resolution ${\hat{H}}_{i}\times {\hat{W}}_{i}$	#Channels ${\hat{C}}_{i}$	#Layers ${\hat{L}}_{i}$
1	Conv3 × 3	224 × 224	32	1
2	MBConv1, *k*3 × 3	112 × 112	16	1
3	MBConv6, *k*3 × 3	112 × 112	24	2
4	MBConv6, *k*5 × 5	56 × 56	40	2
5	MBConv6, *k*3 × 3	28 × 28	80	3
6	MBConv6, *k*5 × 5	28 × 28	112	3
7	MBConv6, *k*5 × 5	14 × 14	192	4
8	MBConv6, *k*3 × 3	7 × 7	320	1
9	Conv1 × 1 & Pooling & FC	7 × 7	1280	1

The input resolution denotes as (${\hat{H}}_{i},{\hat{W}}_{i}$), ${\hat{C}}_{i}$ are output channels [35].

The article "Leaf Recognition Based on Joint Learning Multiloss of Multimodel Convolutional Neural Networks: A Testing for Vietnamese Herb" was published in 2021. Journal: Comput Intell Neurosci.

**Table 6:** Information of the combination dataset (Flavia + Leafsnap + Folio) used in our experiment.

Dataset	Number of classes	Number of leaf images
**Flavia**	32	1907
**Folio**	32	637
**Leafsnap**	184	7552
**Combined dataset (Flavia** **+** **Leafsnap** **+** **Folio) (after merging and removing duplicate classes)**	239	10057

**Table 7:** Some Vietnamese herbal species in our V-Herb database.

Vietnamese herbal species	Scientific names	Vietnamese herbal species	Scientific names
Ắc ó	*Acanthus integrifolius*	Muồng Trâu	*Senna alata*
Bạch HoaXà	*Plumbago zeylanica*	Quỳnh lam	*Gonocaryum lobbianum*
Cà Hai Lá	*Solanum diphyllum*	Ngọc Nữ Biển	*Clerodendrum inerme* (L.) Gaertn
Đinh lăng lá trổ	*Polyscias guilfoylei*	Sâmcaulálớn	*Curculigo capitulata* (Lour.) Kuntze
Hoắc Hương	*Pogostemon cablin*	Vọng cách	*Premna serratifolia*
Lược vàng	*Callisia fragrans*	Xáo tam phân	*Paramignya trimera*

**Table 8:** The accuracy of the U-Net for leaf segmentation.

Dataset	Training set	Validation set	Test set	Accuracy (%)
**Leafsnap**	5173	720	1620	92.21
**Combination dataset (Flavia** **+** **Folio** **+** **Leafsnap)**	5958	1933	2166	93.03

**Table 9:** Results of U-Net segmentation on Flavia and our V-Herb database.

Dataset	Accuracy (%)
Flavia	100
Our V-Herb	98.63

**Table 10:** Performance comparison of various leaf recognition approaches on the Flavia database.

Model	Data augmentation	Accuracy (%)
CNN-LeafNet [17]	Yes	97.90
CNN-data augmentation [40]	Yes	94.69
Inception V3	Yes	99.70
**U-Net** **+** **simple CNN (03 Conv2d)**	No	95.42
	Yes	**99.25**
Simple CNN (03 Conv2d) (without U-Net)	Yes	97.11
**U-Net** **+** **VGG16**	No	**99.50**
VGG16 (without U-Net)	No	98.70
**U-Net** **+** **MobileNet V1**	No	**100**
MobileNet V1 (without U-Net)	No	99.13
**U-Net** **+** **EfficientNet B0**	No	**99.57**
EfficientNet B0 (without U-Net)	No	99.13
**U-Net** **+** **multimodel (proposed)**	No	**100**
Multimodel (proposed) (without U-Net)	No	99.57

**Table 11:** Performance and computation cost comparison of CNNs and our proposed multimodel for leaf recognition on the combination dataset using U-Net.

Models	Accuracy (%)	Computation cost (in average)
VGG16	82.03	0.212
ResNet-50 V2	85.99	0.219
Xception	89.58	0.189
Inception V3	81.35	0.252
Inception-ResNet V2	88.02	0.379
EfficientNet B2	90.58	0.286
EfficientNet B0	89.79	0.235
MobileNet V1	81.64	0.188
**Multimodel (proposed)**	**93.59**	**0.223**

**Table 12:** Performance and computation cost comparison of CNNs and proposed multimodel for leaf recognition on V-Herb database using U-Net.

Models	Accuracy (%)	Computation cost (in average)
Xception	98.86	0.217
Inception-ResNet	98.86	0.382
EfficientNet B2	98.86	0.297
EfficientNet B0	95.71	0.239
MobileNet V1	97.73	0.192
**Multimodel (proposed)**	**98.89**	**0.220**

The article "Leaf Recognition Based on Joint Learning Multiloss of Multimodel Convolutional Neural Networks: A Testing for Vietnamese Herb" was published in 2021. Journal: Comput Intell Neurosci.

**Table 13:** Performance and computation cost comparison of CNNs and proposed multimodel for leaf recognition on V-Herb database with and without U-Net.

Models	Accuracy (%)	
	U-Net-based background removal	Without U-Net
Xception	**98.86**	66.41
Inception-ResNet	**98.86**	82.44
EfficientNet B2	**98.86**	92.37
EfficientNet B0	**95.71**	91.60
MobileNet V1	**97.73**	37.41
**Multimodel (proposed)**	**98.89**	**92.37**

## Data Availability

The data used to support the findings of this study are as follows: public data and private data.
